The article "Isolated olecranon fractures in children affected by osteogenesis imperfecta type I treated with single screw or tension band wiring system: Outcomes and pitfalls in relation to bone mineral density" was published in 2017. Journal: Medicine (Baltimore).

# Isolated olecranon fractures in children affected by osteogenesis imperfecta type I treated with single screw or tension band wiring system: Outcomes and pitfalls in relation to bone mineral density

**DOI:** 10.1097/MD.0000000000006766

**Published:** 2017-05-19

**Authors:** Pietro Persiani, Filippo M. Ranaldi, Jole Graci, Claudia De Cristo, Anna Zambrano, Patrizia D’Eufemia, Lorena Martini, Ciro Villani

**Affiliations:** a Department of Anatomical Sciences, Histological, Forensic Medicine and Locomotive System; b Department of Pediatrics, Sapienza University of Rome, Rome, Italy.

**Keywords:** fracture, olecranon, ORIF, osteogenesis imperfecta, tension band wiring, *Z*-score

## Abstract

The purpose of this study is to compare the results of 2 techniques, tension band wiring (TBW) and fixation with screws, in olecranon fractures in children affected with osteogenesis imperfecta (OI) type I. Between 2010 and 2014, 21 olecranon fractures in 18 children with OI (average age: 12 years old) were treated surgically. Ten patients were treated with the screw fixation and 11 with TBW. A total of 65% of olecranon fractures occurred as a result of a spontaneous avulsion of the olecranon during the contraction of the triceps muscle. The average follow-up was 36 months. Among the children treated with 1 screw, 5 patients needed a surgical revision with TBW due to a mobilization of the screw. In this group, the satisfactory results were 50%. In patients treated with TBW, the satisfactory results were 100% of the cases. The average *Z*-score, the last one recorded in the patients before the trauma, was −2.53 in patients treated with screw fixation and −2.04 in those treated with TBW. TBW represents the safest surgical treatment for patients suffering from OI type I, as it helps to prevent the rigidity of the elbow through an earlier recovery of the range of motion, and there was no loosening of the implant. In analyzing the average *Z*-score before any fracture, the fixation with screws has an increased risk of failure in combination with low bone mineral density.

## 1 Introduction

Osteogenesis imperfecta (OI) is an inherited disease that affects 1:20,000 live births.^[1]^

It is caused by mutations of the α-1 and α-2 chains of type I collagen. Moreover, being the most represented structural protein of the bone and a component of many other extra-skeletal tissues, this disease also presents extra-skeletal manifestations such as hearing loss, blue sclera, dentinogenesis imperfecta, ligamentous laxity, and cardiac anomalies.^[2–5]^

Different classification systems have been introduced for this genetic and clinical heterogeneity. At the moment, 8 different OI types have been classified. These are associated with different genetic mutations.^[6–8]^

The characteristic orthopedic and trauma manifestations of the disease are vertebral fractures, scoliosis, kyphosis, deformities of the long bones, bone fractures from low-energy traumas, or spontaneous avulsions at the level of the tendon insertions.^[9–11]^

Elbow fractures in children are common, equal to 5% to 10% of all pediatric fractures,^[12]^ while the isolated apophyseal detachments of the olecranon represent only 1.7% of all elbow fractures in healthy children.^[13]^ The incidence is higher in children with OI, especially type I.^[14–18]^ Bracq^[14]^ reported that 3 out of 83 olecranon fractures (3.6%) occurred in children with OI. Evans and Graham^[19]^ found that 8 out of 59 olecranon fractures (13.6%) occurred in children with OI. In healthy children, olecranon fractures are classified into 2 main categories: purely apophyseal, which usually affect younger children, and metaphyseal, which affect older children and are characterized by a large metaphyseal fragment adherent to the epiphysis.^[20]^ These fractures can be caused by a direct or indirect mechanism; when they are displaced, in children, they are usually characterized by a single fracture line, with a displacement of >2 mm in about 1/3 of the cases.^[21]^ In children with OI, they are more frequent and are primarily characterized by an indirect mechanism of injury, avulsion fracture, in which the tip of the olecranon can detach, as a consequence of a sudden contraction of the triceps brachial muscle.^[22]^

The purpose of this study is to compare the results of 2 stabilization techniques, tension band wiring (TBW) and fixation with screws, in olecranon fractures in children affected with OI type I.

The treatment for displaced olecranon fractures is always surgery, as this is the only way to reduce the diastasis.^[23,24]^ In the literature, there are no clear indications which surgical technique should be adopted. The most commonly used surgical techniques are fixation with a cannulated screw and osteosynthesis with TBW.^[19,25–28]^ In literature, there are indications that conservatively treated nondisplaced olecranon fractures have excellent long-term results. In healthy patients, displaced fractures have satisfactory results in approximately 78% of cases.^[29]^ With K-wire pinning, or TBW at the level of the olecranon tip, the risk of bone growth arrest for the epiphysiodesis is very rare, given the small diameter of the wire.^[30]^ As for the screw, which has a diameter of 3.5 mm, which is larger than the diameter of a K-wire, the risk of damage to the physis is higher, but still negligible.^[31]^

In this type of fracture, the most common cause for an unsatisfactory result seems to be the limited flexion/extension range of motion (ROM) of the elbow. Considering that the subcutaneous layer is almost nonexistent in the olecranon region, the head of the screw, or the TBW, could cause some discomfort, pain or local skin irritation and, therefore, these fixation devices are removed after stable union of the fracture.

In patients with OI, the immobilization is always brief, compatible with the type of fracture and its healing process, given that the degree of osteoporosis could worsen with prolonged immobilization. Therefore, olecranon fractures are treated surgically and, in the case of a screw fixation osteosynthesis, the elbow is postoperatively immobilized in a long-arm cast extended at 30° for about 20 days, while, with a TBW synthesis, the elbow is placed in a movable brace locked at a 0° to 60 ° extension, then unlocked at a 30° flexion from the first postoperative day, after which complete joint movement is permitted from the second day onward.

## 2 Methods

The present study on human participants was conducted with the approval of the Ethics Committee of Sapienza University of Rome.

At the center of reference for Congenital Osteodystrophies, located in the Department of Pediatrics and the Department of Orthopedics and Traumatology of the Policlinico Umberto I Hospital, around 270 patients are followed. Among these, 18 patients suffering from OI type I with olecranon fractures (10 males and 8 females) were included in our study, for a total of 21 fractures (15 left, 6 right), 3 of these patients had bilateral fractures. All the patients were treated surgically between 2010 and 2014. The age at the time of the fracture was between 9 and 15 years old (average 12 years old). All the patients referred to the Center for Congenital Osteodystrophies were subjected to infusion therapy with neridronate (2 mg/kg) every 3 months, and a bone densitometry with Holologic 4500 (Hologic Inc., Crosby Drive, Bedford, MA) for the *Z*-score quantification every 4 months, in order to verify the bone mineral quality (average value of the *Z*-score in patients with OI type I is 2.38 ± 0.6).^[32,33]^

With regard to the mechanism of the fractures, 13 fractures (65%) occurred spontaneously, caused by an avulsion of the insertion of the brachial triceps muscle, 6 fractures were caused by direct trauma (28.5%), and 2 fractures by indirect trauma (9.5%).

X-ray images in 2 planes were obtained after admission, differentiating the fractures according to the Mayo classification.^[34]^ All the patients were treated surgically at the Orthopedic Department of the Policlinico Umberto I Hospital, by 2 different surgeons, with open reduction and internal fixation with cannulated screws (surgeon: CV) or an osteosynthesis with TBW (surgeon: PP).

The postoperative protocol of the patients treated with TBW called for the placement of a mobile cast with a range of 0° to 60° locked in extension, then unlocked at 30° in flexion from the first postoperative day; once the stitches were removed the tutor was unlocked with full ROM of the elbow, removal of the tutor during the day and a program of an active and passive kinesis of the elbow.

For the patients treated with the screw (Fig. 1), the postoperative protocol involved the placement of an arm-forearm-metacarpal brace, with the elbow extended to 30°; the removal of the brace took place on the 20th postoperative day, with a program of gradual recovery of the ROM of the elbow.

**Figure 1:** Postoperative X-ray shows the osteosynthesis performed using a single cannulated screw.

The postoperative radiographic evaluation was carried out at 20, 60 days, 4, 12 months, and 3 years after the surgery, evaluating a possible loosening of the implant, bone healing, and the presence of periarticular calcification.

The patients were clinically evaluated postoperatively at 20, 60 days, 4, 12 months, and 3 years, considering the pain parameters, joint mobility, joint stability, deformities, and muscle strength.

We decided to exclude all the patients with implant failure from the study, or in need of a surgical revision with TBW, in order to have a uniform sample of patients in our study.

The statistical analysis was performed using the SPSS 20.0 statistical software (IBM Corporation, North Castle Drive, Armonk, NY). The chi-square test was used for the analysis of discrete data and the associations between variables. Comparisons between averages were performed with the *t* test for 2 independent variables and the analysis of variance test for multiple variables.

## 3 Results

The classification of fractures, revealed by the radiographic evaluation, showed 12 type II fractures (57%) and 9 type III fractures (43%), in accordance with the Mayo classification (Fig. 2A and B; Fig. 3).

**Figure 2:** Preoperative X-rays in a male patient (12 years old), showing the fracture/avulsion of olecranon apophysis (Mayo II) in the anterior-posterior (A) and the lateral (B) planes.

**Figure 3:** Fracture/avulsion of olecranon apophysis (Mayo III) in a female patient (14 years old).

A total of 10 olecranon fractures were treated with internal fixation with the screw and the other 11 with TBW (Table 1). The progress was uneventful, 12 out of the 18 patients examined had taken analgesics (paracetamol 500 mg/daily) in the first 7 postoperative days (7 cases treated with the screw and 5 cases treated with TBW) (Table 2).

**Table 1:** Master table showing cases, surgical treatment, limitation in ROM (in grades), complications occurred and pain at 20, 60 days, 4 months, 1, and 3 years after surgery, in relationship to age and fracture type.

**Table 2:** *Z*-scores classification based on different surgical treatment treatment.

### 3.1 On the 20th postoperative day

Pain was present in 10 cases treated with the screw and in 8 cases treated with TBW.

The ROM in 10 fractures treated with the screw showed an average limitation of extension of −75°, while in 11 fractures treated with TBW the average limitation of extension was of −50°.

Upon X-ray examination, all patients showed a good alignment of the bone fragments.

No complications were recorded.

### 3.2 The evaluation on the 60th postoperative day

Pain was present in 5 cases treated with the screw and 3 cases treated with TBW.

The ROM in 10 fractures treated with the screw showed an average limitation of extension of −55°, while in 11 fractures treated with TBW the average limitation of extension was of −15°.

The X-ray imaging of all the patients showed a regular bone callus and no cases of periarticular calcification (Fig. 4A and B).

**Figure 4:** X-rays at 60 days after surgical treatment, performed with tension band wiring, in the anterior–posterior (A) and lateral (B) planes.

Complications: in 2 cases treated with the screw there was a loosening of the implant (Fig. 5A and B), which required a surgical revision and replacement with new screws. We considered these cases as failures, and thus we excluded them from the study.

**Figure 5:** Implant loosening in a male patient (15 years old) treated 60 days before with a single cannulated screw. X-rays in anterior–posterior (A) and lateral (B) planes.

### 3.3 Evaluation on the 4th postoperative month

The pain persisted in 3 cases treated with a screw, one of which showed swelling in correspondence of the screw head, no pain was registered in the patients treated with TBW.

The ROM in all the patients treated with the screw showed an average limitation of extension of −35°, while in all the cases treated with TBW there was an average deficit of extension of less than 10°.

In the X-ray imaging, we observed a regular development of the bone callus in all the patients and no cases of periarticular calcification.

Complications: after radiographic examination, 1 patient had a migration of the screw and underwent a subsequent surgical revision with TBW. This patient also was excluded from the study.

### 3.4 Follow-up at the 12th postoperative month

Pain was absent in all patients.

The ROM indicated an average limitation in extension of −25° in the cases treated with the screw, whereas in patients treated with TBW the ROM was unrestricted.

X-ray imaging showed that all 16 treated elbows had complete bone healing, and there were no cases of periarticular calcification (Fig. 6).

**Figure 6:** X-rays 1 year after surgery, showing the excellent outcome in fracture healing.

Complications: 2 patients treated with screws reported an olecranon refracture with implant migration, which required a surgical revision with TBW. These patients were therefore excluded from the study.

### 3.5 Evaluation 3 years after surgery

Pain was absent in all patients.

All the patients had a full pronation/supination ROM of the forearm, none of them presented with angular deviations of the elbow; nevertheless, an average limitation of extension of −15° persisted in patients treated with the screw, while in all the patients treated with TBW the flexion–extension recovery was full.

X-ray imaging of all the elbows showed complete bone healing, no cases of periarticular calcification and no cases of implant migration.

The average *Z*-score, the last one recorded in the patients before the trauma, was −2.53 in patients treated with the screw and −2.04 in those treated with TBW. The *Z*-score is connected to the specific surgical treatment, since bone screws may have a weaker grip in the osteoporotic bone, thus resulting in a worse compression and synthesis of the fracture, compared to the mechanical effect obtained with the TBW.

## 4 Discussion

In the studied series, 65% of olecranon fractures, in children with OI, occurred with a nontraumatic avulsion of the olecranon's tip while contracting the triceps muscle. In addition, these patients are at high risk with a 70% chance of suffering a similar contralateral fracture or refracture.

Ogden^[35]^ observed that, with regard to healthy children, in the metaphyseal portion of the proximal ulna, the subchondral bone is well represented, and this feature predisposes them to a peculiar type of avulsion fracture, characterized by the detachment of an apophyseal fragment together with a thin layer of metaphyseal bone can occur. This pattern, however, is very rare and occurs in children under the age of 10 years.

Wilkins^[20]^ has instead suggested that apophyseal avulsion fractures of the olecranon rarely occur in healthy children, because the expansions of the triceps tendon have their insertion on the metaphysis and distally to the physis.

Children with OI are more predisposed to this type of fracture, compared to healthy children, since the combination of the fragility of the bone adjacent to the physis of the olecranon, and the increased laxity of the expansions of the triceps, could make the olecranon apophysis more vulnerable to avulsions in children suffering from this disease.^[25]^

Upon examination, these fractures are characterized by tenderness and swelling in the proximal part of the elbow. Sometimes, in children with OI type I, the general characteristics of the disease may be blurred. OI type I is, in fact, characterized by mild osteopenia, absence of deformity of the long bones, and normal stature. For this reason, it is not always easy to make a definite diagnosis of a fracture due to OI, and many of the olecranon fractures in children with OI Type I go unrecognized or undiagnosed. In literature, it has been described as a differential diagnosis with a fracture due to abuse.^[9]^

In our case, at the time of the fracture, all the patients were already in the care of the doctors of the Center for Congenital Osteodystrophies, located in the Department of Pediatrics of our university hospital (Policlinico Umberto I) and, therefore, already had a diagnosis of OI with specific genetic typing.

In literature, several authors ^[14,17,25]^ described that the olecranon fracture is one of the “typical fractures” of OI, since the moment of birth. The treatment is always surgical and can vary from transosseous suture, in neonatal age and early childhood, to internal fixation with screw or TBW in children older than 8 years of age.

It is difficult to make a detailed comparison and review of the literature on this subject, given the rarity of OI and the even more rare incidence of olecranon fractures in patients with a proven and documented diagnosis of OI type I. However, when comparing our study with other studies that address the same subject, we observed that TBW is considered a first choice treatment in olecranon fractures for patients with OI.

The incidence of refracture or new contralateral olecranon fracture is highly likely in patients with OI and other studies confirm this fact.^[25,27]^ In our study, it occurred in 3 out of 18 patients (17%).

With regard to the risk of growth arrest due to the involvement of the physis during the synthesis procedure, although our study did not register any cases in which this type of problem had occurred by the end of follow-up, the treatment with TBW is preferable compared to that with the screws because of a lower pin diameter. However, the ossification core of the olecranon's apophysis, which manifests itself around 9 years of age, contributes to a very small percentage of the total longitudinal ulnar growth. Therefore, a growth arrest in this core is very rare and insignificant, especially considering that, in our specific case, the average age of the patients (12 years old) is higher than in the period in which this core is more at risk.

The osteosynthesis with TBW, in addition to exploiting the principle of TBW,^[36]^ allows early mobilization, preventing elbow stiffness, and a more rapid recovery of the ROM in comparison to the treatment of internal fixation with the cannulated screw. The objective of early mobilization, in children with OI, is critical in order to not aggravate the degree of osteoporosis from which they are suffering. One disadvantage of TBW, not encountered in our study but described by other authors,^[27]^ is the frequent need for implant removal, as it may cause local irritation subcutaneously. This removal causes a high risk for a refracture of the olecranon in children with OI.

Other surgical techniques, used to treat this type of fractures in patients with OI type I, are not described in literature. However, Rath et al^[37]^ describe the transosseous suture for the fixation of fragments as an alternative method, which has given excellent results in healthy pediatric patients.

Moreover, the cases treated with the screw, in which there had been a traumatic implant loosening (equal to 30% of the sample), had a lower average *Z*-score of 2.53 at the time of the trauma. Therefore, the failures observed in our study depended on this characteristic. This is confirmed by the positive results obtained with patients treated with TBW who, although also suffering from severe osteoporosis, benefited from a synthesis that was not conditioned by their bone quality, which enabled them to resume elbow function more quickly, with a reduction of immobilization time that, if extended, would have resulted in a deterioration in the degree of osteoporosis.

In patients with an olecranon apophysis fracture, due to an isolated avulsion by contraction of the triceps without trauma, a differential diagnosis with OI type I should be considered.

In relation to the treatment, the failure of the osteosynthesis with cannulated screw can be traced to an inadequate adhesion of the implant to the osteoporotic bone of patients with OI type I. In addition, a low *Z*-score value must be considered as a predisposing factor for failures or complications.

Patients suffering from OI require short recovery times, with immobilizations that are not too prolonged in time, which could otherwise worsen the underlying osteoporosis in this pathology. For this reason, TBW seems to be an adequate means of osteosynthesis for these fractures, as the system's hold does not require a strong grip within the bone, thereby reducing the failure rate. At the same time, TBW allows patients to mobilize the elbow joint more rapidly, taking advantage of the mechanical principle of the tie rod, according to which the force applied to the elbow flexion is transformed into compressive force, which promotes a rapid functional recovery. In addition, with this treatment it is unlikely for the physis to be injured, as the diameter of the pins with which the TBW is done is smaller than that of a screw. However, because of the risk of local skin irritations, due to the chronic friction between the implant and the skin, the removal of the TBW is recommended, although early removal can lead, with high probability, to a refracture in the same area.

In conclusion, in our study, the safest treatment for fractures of the olecranon in children with Type I OI appears to be the fixation with TBW, because it showed the best results in terms of joint function recovery time, with a lower incidence of complications and pain, which allowed patients to have a significant recovery of their quality of life.
